RETRACTED

# HSP70 Domain II of *Mycobacterium tuberculosis* Modulates Immune Response and Protective Potential of F1 and LcrV Antigens of *Yersinia pestis* in a Mouse Model

**DOI:** 10.1371/journal.pntd.0003322

**Published:** 2014-12-04

**Authors:** Lalit Batra, Shailendra K. Verma, Durgesh P. Nagar, Nandita Saxena, Prachi Pathak, Satish C. Pant, Urmil Tuteja

**Affiliations:** 1 Microbiology Division, Defence Research & Development Establishment, Gwalior, India; 2 Pharmacology and Toxicology Division, Defence Research & Development Establishment, Gwalior, India; University of Notre Dame, United States of America

## Abstract

No ideal vaccine exists to control plague, a deadly dangerous disease caused by *Yersinia pestis*. In this context, we cloned, expressed and purified recombinant F1, LcrV antigens of *Y. pestis* and heat shock protein70 (HSP70) domain II of *M. tuberculosis* in *E. coli*. To evaluate the protective potential of each purified protein alone or in combination, Balb/C mice were immunized. Humoral and cell mediated immune responses were evaluated. Immunized animals were challenged with 100 LD_50_ of *Y. pestis* via intra-peritoneal route. Vaccine candidates *i.e.*, F1 and LcrV generated highly significant titres of anti-F1 and anti-LcrV IgG antibodies. A significant difference was noticed in the expression level of IL-2, IFN-γ and TNF-α in splenocytes of immunized animals. Significantly increased percentages of CD4+ and CD8+ T cells producing IFN-γ in spleen of vaccinated animals were observed in comparison to control group by flow cytometric analysis. We investigated whether the F1, LcrV and HSP70(II) antigens alone or in combination can effectively protect immunized animals from any histopathological changes. Signs of histopathological lesions noticed in lung, liver, kidney and spleen of immunized animals on 3^rd^ day post challenge whereas no lesions in animals that survived to day 20 post-infection were observed. Immunohistochemistry showed bacteria in lung, liver, spleen and kidney on 3^rd^ day post-infection whereas no bacteria was observed on day 20 post-infection in surviving animals in LcrV, LcrV+HSP70(II), F1+LcrV, and F1+LcrV+HSP70(II) vaccinated groups. A significant difference was observed in the expression of IL-2, IFN-γ, TNF-α, and CD4+/CD8+ T cells secreting IFN-γ in the F1+LcrV+HSP70(II) vaccinated group in comparison to the F1+LcrV vaccinated group. Three combinations that included LcrV+HSP70(II), F1+LcrV or F1+LcrV+HSP70(II) provided 100% protection, whereas LcrV alone provided only 75% protection. These findings suggest that HSP70(II) of *M. tuberculosis* can be a potent immunomodulator for F1 and LcrV containing vaccine candidates against plague.

RETRACTED

## Author Summary

Efforts are in progress by various scientific groups towards the development of plague vaccines. However, lack of better understanding about the *Y. pestis* infection mechanisms and pathogenesis prevents the development of an effective vaccine. In our effort to develop a more efficacious plague vaccine, we evaluated the role of HSP70 (domain II) of *M. tuberculosis* in formulation with the F1 and LcrV subunits of *Y. pestis* vaccine candidates. It is well documented that the F1 and LcrV alone does not always provide complete protection whereas a mixture of the F1+LcrV provides 100% protection in mouse model but poorly protect African green monkey models. In this study, LcrV provided 100% protection in formulation with HSP70(II) whereas LcrV alone could provide only 75% protection in *Y. pestis* challenged mice. Two another combinations *i.e.*, F1+LcrV and F1+LcrV+HSP70(II) also provided 100% protection whereas HSP70(II) or F1 alone failed to protect. HSP70(II) also modulated cellular immune response as the significantly elevated levels of IL-2, IFN-γ, TNF-α and IFN-γ secreting CD4+/CD8+ T cells were noticed in spleen of F1+LcrV+HSP70(II) group in comparison to the F1+LcrV group. These findings describe the role of HSP70(II) and propose future perspectives for development of new generation plague vaccine.

## Introduction

Plague caused by *Y. pestis* (a Gram negative bacterium) is a zoonotic infectious disease that has profoundly affected the course of history [1], [2] and troubles human populations, leading to millions of deaths. According to the World Health Organization (WHO), plague has been classified as a re-emerging infectious disease [3]. Rodents are the reservoirs for *Y. pestis* and the fleas transmit the bacteria from rodent to rodent. Infected fleas also transmit bubonic plague, the most common form of the disease from rodents to humans [4]–[6]. Humans are infected accidently after bites from fleas having *Y. pestis*, by direct contact with blood and tissues of infected animals, or by direct aerosol transmission. The aerosol transmission develops lethal pneumonic plague. The intentional aerosolization of *Y. pestis* in human population is the main concern of bioterrorism [7]. Plague can be treated with antibiotics at early stage. It has been reported that antibiotic-resistant strains of *Y. pestis* bacilli have been isolated in Madagascar and Mongolia [8], [9] and showed naturally acquired multi-drug-resistant variants of *Y. pestis* [10]. These studies suggest that there is an urgent need to develop an effective vaccine that can provide long term protection and to counter the drug resistant variants of *Y. pestis*.

RETRACTED

Administration of live attenuated *Y. pestis* vaccine provides protection against plague in animal models [11], [12]. These live attenuated plague vaccines are accessible in some countries, like Russia [13]; however, in the United States and Europe, these vaccines have never been licensed most probably due to several risk factors associated with the use of live-attenuated or whole cell killed vaccine in terms of side effects and administration of numerous antigens from live/killed vaccines [13]–[16]. Hence it is very much essential to develop new generation vaccines. Earlier studies using F1/LcrV-based vaccines that protect mouse models and cynomolgus macaques against aerosolized *Y. pestis* but they confer poor and inconsistent protection in African Green monkey models [17], [18]. Further in order to improve the efficacy of F1/LcrV-based vaccines, several approaches are in progress. Amongst these, genetically modified antigens [19], use of alternate adjuvants [20], [21] and delivery systems [22], [23] are very important as these approaches are certainly promising. It is noteworthy to mention that F1-negative *Y. pestis* strains persists [24], and LcrV variants of *Y. pestis* may pose serious challenge for any vaccine with respect to cross-protection [25], [26]. With this background, one possible strategic approach could be the inclusion of additional antigen/s that might play the role of an immunomodulator/s or and an immunoregulator/s to augment the immune response in the subunit vaccine preparation to encounter the possible disease threat.

It has been established in the recent studies that subunit vaccines protect mouse models by inducing F1/LcrV-specific humoral immune response; however, to achieve complete protection cell mediated immune response mainly relies on the type-1 cytokines *i.e.*, IFN-γ and TNF-α [27]–[29]. These findings suggest that the efficacy of subunit vaccines might be improved if they induce *Y. pestis*-specific IFN-γ and TNF-α secreting memory T cells in addition to F1/LcrV-specific humoral immunity. In this scenario, it would be highly valuable to modulate the immune response of F1/LcrV antigens to create an effective plague vaccine. In context to this, the heat shock proteins70 are well documented to augment the immune response for the development of vaccine initiatives [30]–[35]. It has been proven that the role of HSP70(II) in stimulating effective T-cell responses [36] to pathogen-specific antigens. As reported earlier, HSP70(II) of *M. tuberculosis* is known to play crucial role in antigen processing and presentation by MHCs [37]. Huang *et al*. [36] demonstrated the role of fusion construct using ovalbumin-HSP70, domain II [38], amino acid (161–370) of HSP70 from *M. tuberculosis*, is sufficient to elicit ovalbumin specific CD8+ cytotoxic T lymphocytes (CTLs).

RETRACTED

Here, in order to evaluate the HSP70(II) as an immunomodulator, we have cloned *caf1* and *lcrV* genes of *Y. pestis* and *hsp70(II)* gene of *M. tuberculosis*. The encoding proteins were expressed in *E. coli* and purified upto homogeneity. In order to evaluate the protective efficacy, Balb/C mice were immunized with purified proteins F1, LcrV, and HSP70(II) alone or in combinations. Humoral and cell mediated immune responses were also evaluated. Immunized animals were challenged with 100 LD_50_ of *Y. pestis* via intra-peritoneal route. Significantly high IgG response was observed in the sera of immunized mice with F1 and LcrV alone or in combinations. Three combinations *i.e.*, LcrV+HSP70(II), F1+LcrV and F1+LcrV+HSP70(II) provided 100% protection. HSP70(II) modulated cellular immune response as the significantly elevated levels of IL-2, IFN-γ, TNF-α and IFN-γ secreting CD4^+^/CD8^+^ T cells were noticed in spleen of F1+LcrV+HSP70(II) group in comparison to the F1+LcrV group. HSP70(II) also increased protective efficacy of LcrV from 75 to 100%. We also performed the histopathological studies to examine the liver, spleen, lung and kidney tissues from immunized animal groups that were intraperitoneally infected with virulent *Y. pestis* at 3^rd^ and 20^th^ day post infection. *Y. pestis* localization in tissues was also examined by immunohistochemistry using fluorescent microscopy.

## Materials and Methods

### Ethics statement

Institutional Animal Ethics Committee (IAEC) of Defence Research and Development Establishment “approved” all the protocols for experiments conducted using mice wide registration number 37/Go/C/1999/CPCSEA and Institutional Biosafety committee (IBSC) wide protocol no: IBSC/21/MB/UT/12 as per the institutional norms. The principles of good laboratory animal care were followed all through the experimental process. The mice were maintained in accordance with recommendations of committee for the purpose of control and supervision of experiments on animals, Govt. of India.

### Bacterial strains and reagents

A virulent strain of *Y. pestis* (clinical isolate, designated as S1) recovered from a patient during a sporadic outbreak of primary pneumonic plague occurred in Northern India in 2002 [39], [40] was used for challenging experiments. Frozen stock of *Y. pestis* was streaked on Brain Heart Infusion (BHI) agar plate and incubated at 28°C for 48 h. A single colony from BHI agar plate was further inoculated in 5 ml of BHI broth and grown at 28°C for 48 h and the colonies (CFU/ml) were counted. All live *Y. pestis* cultures and animal experiments were performed in BSL-3 facility, DRDE, Gwalior. *E. coli* host strain BL21 (DE3) and DH5α were purchased from Invitrogen, USA. The expression vector pET 28a^+^ was from Novagen, USA.

RETRACTED

### Cloning of *caf1, lcrV* and *hsp70(II)* genes in pET vector

*Y. pestis*, S1 strain was grown in BHI broth at 28°C and the genomic DNA was isolated by DNeasy Blood and Tissue kit (Qiagen, USA). The genomic DNA of *M. tuberculosis* was a generous gift from DFRL, Mysore, India. The genes *caf1* and *lcrV* of *Y. pestis* and *hsp70(II)* of *M. tuberculosis* were amplified by polymerase chain reaction (PCR). The details of used oligos in this study are given in Table 1. The individual amplicon was ligated into pET28a vector using compatible restriction sites. The individual ligated product was transformed into chemically competent cells of *E. coli* host strain DH5α and the positive clones were selected on Luria Bertani (LB) agar plates supplemented with kanamycin (50 µg/ml). The plasmid DNA was isolated by using QIAprep Spin Miniprep Kit (Qiagen, USA) from overnight grown culture corresponding to individual clone.

**Table 1:** List of oligos used for Cloning of *caf1, lcrV* and *hsp70(II)* genes in pET28a^+^ vector.

Gene	Oligos	Restriction sites	Amplicon Size (bp)	Accession No.
*caf1*	F-5′-atacc**atg**ggcATGAAAAAAATCAGTTCCGTTATCG-3′	*Nco* I	513	AF074611.1
	R-5′-atactcgagTTGGTTAGATACGGTTACGGTTACAG-3′	*Xho* I		
*lcrV*	F-5′-cat**atg**ATTAGAGCCTACGAACAAAAC-3′	*Nde* I	981	NC003131.1
	R- 5′-gtcgacTCATTTACCAGACGTGTCATCTAG-3′	*Sal* I		
*hsp70(II)*	F-5′-atacc**atg**ggcGAGAAGGAGCAGCGAATCCTG-3′	*Nco* I	630	CP002992.1
	R-5′-atactcgagCGGGGTAACATCAAGCAGCAG-3′	*Xho* I		

Homologous nucleotide sequences of *caf1, lcrV* and *hsp70(II)* in capital case and the engineered sequences (ata) at the 5′ ends are shown in small case. The in-frame initiator codon in the forward primer is shown in bold and the compatible restriction sites are underlined.

### Expression and purification of recombinant F1, LcrV and HSP70(II) proteins

In order to express the recombinant antigens, *E. coli* host strain BL21 (DE3) cells were transformed with individual recombinant construct corresponding to *caf1, lcrV* and *hsp70(II)*. The positive transformants were selected on LB agar plates containing kanamycin (50 µg/ml) and were inoculated into 5 ml of LB medium with kanamycin and grown at 37°C. Cultures at logarithmic phase (OD_600_ ∼0.75) were induced with 1 mM isopropylthiogalactoside (IPTG) and grown for 3 h. The cultures were pelleted and the cells were lysed in sample buffer and analyzed by SDS–PAGE. The recombinant F1 was purified using Ni-NTA column (Qiagen, USA) under denaturing conditions using 8 M urea following our earlier standardized protocol [41]. Recombinant LcrV and HSP70(II) were purified in native conditions using Ni-NTA column according to the manufacturer's instruction. The purity of the recombinant proteins was analysed by SDS-PAGE and confirmed through western blot using monoclonal antibodies specific for 6X-his tag (Qiagen, USA). The purified proteins F1, LcrV and HSP70(II) were separated by SDS-PAGE and analysed by Western blot using hyper immune sera at 1∶1000 dilution. The purified proteins were dialyzed and concentrated by using Amicon ultra centrifugal filter devices (Millipore) and the concentrations were estimated by Bradford method [42]. The endotoxin levels were measured by Limulus Amoebocyte Lysates (LAL) QCL-1000 kit (Cambrex Biosciences, USA) as per the manufacturer's protocol.

RETRACTED

### Immunization of mice

Immunogenicity of recombinant proteins alone or in combination and protection of immunized mice against virulent *Y. pestis* (S1 strain) was evaluated in 6–8 week old female Balb/C mice. The animals were taken in three batches and divided into 8 groups/batch (8 mice/group) *i.e.*, Control group; HSP70(II) group; F1 group; LcrV group; F1+HSP70(II) group; LcrV+HSP70(II) group; F1+LcrV group and F1+LcrV+HSP70(II) group (Figure 1d [A]). The animals of batch-I were used for evaluation of IgG antibody response and protection studies against *Y. pestis* challenge; batch-II for evaluation of cell mediated immune response (cytokine profiling and the estimation of CD4^+^ and CD8^+^ T cells) and batch-III for histopathological/immunohistochemical studies. All the animal groups were immunized subcutaneously with 10 µg/mouse of each purified corresponding antigen/s as designated by their group name in formulation with aluminium hydroxide gel (0.35% in sterile phosphate buffer saline, PBS). The animals of control group were injected with PBS only. The prime dose was given on day 0 followed by two boosters on day 14 and 21. Blood was collected after first and second booster from each group on day 0, 21 and 28, sera were separated for IgG antibody response (Figure 1d [B]).

**Figure 1:** a. Schematic diagram of three recombinant vaccine candidates; F1, LcrV and HSP70(II) showing the histidine tag and orientation of the open reading frame. **b**. 16% SDS-PAGE analysis of F1 protein expression [**A**]. 12% SDS–PAGE analysis of LcrV [**B**] and of HSP70(II) domain II of *M. tuberculosis* protein expression in *E. coli* [**C**]. The panels depict protein molecular mass marker (lane M), and Coomassie-stained polypeptide profiles of *E. coli* lysates un-induced (lane U) and induced with IPTG (lane I). The arrows at the right of the panels indicate the position of expressed recombinant proteins. **c**. SDS-PAGE analysis of purified F1 [**A**], LcrV [**B**] and HSP70(II) domain II of *M. tuberculosis* [**C**] metal affinity chromatography using Ni-NTA column. Each purified protein (3 µg/well) was analysed on SDS-PAGE. **d**. The humoral and cell mediated immune responses, protective potential and histopathological examinations of F1 and LcrV from *Y. pestis* with or without HSP70(II) of *M. tuberculosis* were evaluated in a mouse model. [**A**] Balb/C mice (8/group) were immunized with plague vaccine candidates with HSP70(II) as an immunomodulator in formulation aluminium hydroxide gel. [**B**] Schematic representation of immunization schedule following challenge experiments.

RETRACTED

### Evaluation of humoral immune response

#### IgG titer

Titers of anti-F1 and anti-LcrV antibodies were assayed in the hyper-immune sera collected after first and second boosters on day 14 and 28 using indirect ELISA. Briefly, ELISA plates (Nunc-Immuno Plate, Denmark) were coated with each individual antigen *i.e.*, F1 and LcrV (0.1 µg/well) in 0.05 M carbonate-bicarbonate buffer, pH 9.6 for overnight at 4°C. The plates were washed thrice with PBS containing 0.05% tween 20 (PBS-T) and blocked with 200 µl of 3% bovine serum albumin (BSA) in PBS for 2 h at 37°C. For anti-F1 antibody, test sera from animal groups *viz*; control, F1, F1+HSP70(II), F1+LcrV F1+LcrV+HSP70(II) after first and second booster were serially diluted (twofold) in PBS starting from 1∶1000 to 1∶128000 and 1∶4000 to 1∶512000 respectively. For anti-LcrV antibody, test sera from animal groups *viz*; control, LcrV, LcrV+HSP70(II), F1+LcrV F1+LcrV+HSP70(II) after first and second booster were serially diluted (twofold) in PBS starting from 1∶1000 to 1∶256000 and 1∶5000 to 1∶1280000 respectively. The sera were taken in triplicate wells (100 µl/well) and incubated for 1 h at 37°C. The ELISA plates were washed five times with PBS-T. Rabbit anti-mouse (IgG) antibodies conjugated to horseradish peroxidase, HRP (Sigma, USA) were diluted 1∶20000 in PBS, added to wells and incubated for 1 h at 37°C. After five washings, the plates were incubated with o-phenylenediamine dihydrochloride as substrate (100 µl/well) for 10 min. The reaction was stopped by 2N H_2_SO_4_ and the absorbance was read at 490 nm in an ELISA reader (Biotek Instruments, USA).

### Evaluation of cell mediated immune response

#### Cytokine profiling

Three mice from all the eight groups of batch-II were randomly selected, sacrificed and their spleens were removed aseptically. The cytokine estimation was performed using the method published earlier [43]. Briefly, single cell suspension of splenocytes was prepared by maceration of spleens. The splenocytes from each mouse (1×10^6^ cells/well) were suspended in a 24-well tissue culture plate in triplicates. The cultures were stimulated with particular antigen/s alone or in combination (5 µg/ml each antigen) corresponding to their designated groups or Concanavalin A (Con A, 5 µg/ml; Sigma, USA). The culture supernatants from the wells were collected after 48 h. The expression of cytokines *i.e.*, TNF-α, IFN-γ, IL-2, IL-4 and IL-10 were measured by ELISA using BD OptEIA Kit, (BD Biosciences, USA) according to the manufacturer's instructions. The levels of cytokines were determined with the help of standard curves generated using recombinant cytokines (BD Biosciences, USA) and presented as picograms per millilitre (pg/ml).

RETRACTED

#### Flow cytometric analysis of IFN-γ producing CD4+ and CD8+ T cells

Three mice from all the eight groups of batch-II were randomly selected, sacrificed and splenocytes were prepared and suspended as described earlier. For estimating frequency of antigen-specific IFN-γ secreting CD4 and CD8 population, splenocytes were stimulated with particular antigen/s alone or in combination (5 µg/ml each antigen) corresponding to their designated groups. Anti-mouse CD28 antibody was used for costimulation and Brefeldin A (1.0 µg/well, Golgistop) was added to prevent secretion of cytokines. Following 6 h incubation, cells were treated with FACS lysing solution (BD Biosciences) to lyse the RBCs and then splenocytes were washed with FACS staining buffer (BD Biosciences). Later, cells were subjected to surface staining with FITC labelled rat anti-Mouse CD4 and CD8a monoclonal antibodies (BD Biosciences) for 30 min at room temperature in dark. After permeabilization with BD cytofix/cytoperm Kit (BD Biosciences), cells were treated with PE labelled rat anti-mouse IFN-γ monoclonal antibodies (BD Biosciences) for 30 min at room temperature in dark. Unstimulated specimens were used to measure spontaneous cytokine production. Stained cells were washed with cold PBS and then acquired in Becton Dickinson FACS Calibur Flow-Cytometer. A total of 10,000 live events, according to forward and side-scatter parameters were accumulated and analyzed using CellQuest Pro software.

### Protection studies

In order to determine the protective efficacy, all the immunized animals of batch-I were challenged with virulent *Y. pestis* (S1 strain) with 100 LD_50_ (1 LD_50_  = 10^3^ CFU/mouse) by intraperitoneal route on day 60 after the prime vaccination. The virulence and the LD_50_ of *Y. pestis* (S1 strain) have been characterized earlier by our group [40]. Survival of the animals was monitored for 30 days after challenge (Figure 1d [B]). Infection was confirmed by isolation and growth of *Y. pestis* on blood agar plate from the different organs viz; lung, liver, spleen and kidney of dead animals.

RETRACTED

### Histopathological studies

For histopathology, all the immunized animals of batch-III were challenged as described earlier for protection studies. At 3^rd^ day post infection, three mice in each group were sacrificed and the organs *viz*: lung, liver, spleen and kidney were collected. The tissues were placed into 10% neutral buffered formalin, dehydrated in serial alcohol gradient (70, 80, 90 and 100%), cleared with xylene, infiltrated in wax (Leica TP-1020) and embedded in paraffin [44]. Three animals from each survived group *i.e.*, LcrV; LcrV+HSP70(II); F1+LcrV and F1+LcrV+HSP70(II) on day 20 post infection and three naive control animals (neither immunized nor challenged) were sacrificed. As described above, their tissues were removed and fixed in 10% neutral buffered formalin for paraffin block preparation. Various sections of 4–5 µm thickness were prepared (Microm HM-360) and stained with haematoxylin and eosin (HE) and analysed under light microscope (Leica, DMLB).

### Immunohistochemistry

For the presence of *Y. pestis*, the tissues sections were also used for immunohistochemical studies [45]. Briefly, sections were deparaffinised, cleared with xylene and rehydrated. The tissues sections were washed with PBS and subjected to antigen-retrieval by boiling in 0.1 M citrate buffer [pH 6.0] for 10 min. The sections were then incubated with 3% H_2_O_2_ in methanol for 10 min to block the endogenous peroxidase activity and blocked with 5% skimmed milk in PBS for 2 h. The tissue sections were incubated with mouse anti-F1 antibody at 1: 1000 dilutions for overnight at 4°C. After three washings with PBS (each for 5 min), sections were incubated with FITC-labelled rabbit anti mouse secondary antibody for 1 h at room temperature and again washed thrice with PBS. The tissue sections were cover slipped using PBS/glycerine (1∶3) and observed under fluorescence microscope (Leica, Germany) using Leica application suit software.

### Statistical analysis

Statistical comparisons for IgG titers, cytokine levels and IFN-γ secreting CD4^+^ and CD8^+^ T cells were performed. Analysis was done using SigmaStat 3.5, by one way ANOVA, All Pairwise Multiple Comparison Procedure (Fisher LSD Method). *P<0.05; ** P<0.01; *** P<0.001; ^#^ P<0.001. Gehan-Breslow-Wilcoxon test was used to compare the protective potential against *Y. pestis* infection amongst different vaccinated. Survival curve analysis (percentage survivals) was done by Kaplan Meier's method (****P<0.0001, ***P<0.001).

RETRACTED

### Accession numbers

The genes *caf1, lcrV* of *Yersinia pestis* and *hsp70(II)* of M. tuberculosis were used in this study for primer designing under the NCBI accession *AF074611.1*, *NC003131.1* and *CP002992.1* respectively. The gene sequences to *lcrV* and *caf1* from *Y. pestis* (*S1 strain*, an Indian clinical isolate) were submitted to GenBank at NCBI under the Accession No. *KF682423* and *KF682424* respectively.

## Results

### Cloning, expression and purification of recombinant F1, LcrV and HSP70(II)

The genes *caf1* (513 bp) encoding F1 (∼17 kDa), *lcrV* (981 bp) encoding LcrV (∼38 kDa) of *Y. pestis* and *hsp70(II)* (630 bp) encoding a domain II of HSP70 (∼23 kDa) of *M. tuberculosis* were cloned in the pET 28a vector. The in-frame and the orientation of the cloned genes were confirmed by nucleotide sequencing (Chromous, Biotech, India). The schematic diagram (Figure 1a) of the three recombinant proteins represents the location of histidine tag and orientation of open reading frame. The nucleotide sequences to *lcrV* and *caf1* genes from *Y. pestis* (*S1 strain*, an Indian clinical isolate) were submitted to GenBank at NCBI under the Accession No. *KF682423* and *KF682424* respectively. The recombinant constructs corresponding to F1, LcrV and HSP70(II) were transformed in BL-21 (DE3). Small-scale cultures of the positive clones were subjected to IPTG induction to identify clones capable of expressing the predicted size of recombinant proteins. The expression profile of recombinant proteins F1, LcrV and HSP70(II) were analysed by SDS-PAGE. A typical induction experiment comparing the polypeptide SDS-PAGE profiles of un-induced and IPTG-induced cultures for F1, LcrV and HSP70(II) are shown in Figure 1b [A], [B] and [C] respectively.

To facilitate the purification of the recombinant proteins, the constructs were designed to carry the 6X-His tag either at N-terminus or C-terminus. Lysis under native conditions revealed the association of recombinant F1 with the pellet fraction, demonstrating that the F1 protein was insoluble. However, LcrV and HSP70(II) were associated with supernatant fractions, demonstrating that LcrV and HSP70(II) were soluble. The purification of the LcrV and HSP70(II) was carried out in native conditions, however, F1 carried out by solubilizing in 8 M urea and purified by Ni-NTA affinity chromatography. The purified recombinant proteins were analysed by SDS-PAGE as shown in Figure 1c. The proteins *i.e.*, F1 [A]; LcrV [B] and HSP70(II) [C] observed to be almost pure. The concentrations of the purified proteins were estimated and the yield of F1, LcrV and HSP70(II) was 14, 20 and 25 mg/L of shake flask cultures respectively. In a western blot experiment, anti-histidine antibody recognized these proteins corresponding to their molecular weights. Immunoblot with hyper immune sera against F1, LcrV and HSP70(II) recognized the corresponding proteins (Figure S1). The endotoxin content performed by LAL assay of purified protein was less than 5EU per 25 µg of each purified protein.

RETRACTED

### Humoral immune response elicited by vaccine formulations

To evaluate the IgG endpoint titers in all the vaccinated groups, total IgG were measured to F1 and LcrV in sera samples collected seven days after first and second boosters respectively. The cut-off value for the assays was calculated as the mean OD (+2 SD) from sera of control group assayed at 1∶100 dilution. The endpoint IgG titers were calculated as reciprocal of the highest serum dilution giving an OD more than the cut-off.

#### F1-specific IgG

The IgG endpoint titer to F1 was 6.4×10^4^ in sera from F1+LcrV+HSP70(II) group whereas it was 3.2×10^4^ from F1; F1+HSP70(II) and F1+LcrV groups after first booster. The IgG endpoint titer after second booster was 2.56×10^5^ from F1+LcrV+HSP70(II) group and 1.28×10^5^ from F1+LcrV group. However, it was 1.28×10^5^ from F1+HSP70(II) group and only 6.4×10^4^ from F1 group (Figure 2A). HSP70(II) significantly increased the IgG response in the immunized groups *i.e.*, F1+HSP70(II) and F1+LcrV+HSP70(II) in comparison to F1, and F1+LcrV groups respectively.

**Figure 2:** Measurement of serum IgG antibody titers in immunized Balb/C mice. [A] Sera collected after first booster (14^th^ day) and second boosters (21^st^ day) from immunized groups (F1, F1+HSP70(II), F1+LcrV, F1+LcrV+HSP70(II)) were measured for F1-specific IgG by indirect ELISA. [B] Determination of LcrV-specific serum IgG antibody titer in the sera from immunized groups (LcrV, LcrV+HSP70(II), F1+LcrV, F1+LcrV+HSP70(II)). Data are represented in mean antibody titers with SD of eight Balb/C mice in each group. The cut-off value for the assays was calculated as the mean OD (+2 SD) from sera of control group assayed at 1∶100 dilution. Serum endpoint IgG titers were calculated as the reciprocal of the highest serum dilution giving an OD more than the cut-off. Analysis was done by one way ANOVA, All Pairwise Multiple Comparison Procedure (Fisher LSD Method). ** P<0.01; *** P<0.001; ^#^ P<0.001.

#### LcrV-specific IgG

The IgG endpoint titer to LcrV was 1.28×10^5^ in sera from F1+LcrV+HSP70(II) and F1+LcrV groups whereas it was 3.2×10^4^ from LcrV group and 6.4×10^4^ from LcrV+HSP70(II) group after first booster. The IgG endpoint titer after second booster was 6.4×10^5^ from F1+LcrV+HSP70(II) group and 3.2×10^5^ from F1+LcrV group. However, it was 3.2×10^5^ from LcrV+HSP70(II) group and 1.6×10^5^ from LcrV group (Figure 2B). HSP70(II) significantly increased the IgG response in the immunized groups *i.e.*, LcrV+HSP70(II) and F1+LcrV+HSP70(II) in comparison to LcrV and F1+LcrV groups respectively.

RETRACTED

### Cell mediated immune response elicited by vaccine formulations

#### Cytokine estimation

Cytokine profiles of all immunized animal groups were determined by estimating the levels of IL-2, IL-4, IL-10, IFN-γ and TNF-α in supernatants of splenocytes stimulated with specific antigen/s. Significantly high (***p<0.001) expression levels of IL-2 (Figure 3A), and TNF-α (Figure 3C) were noticed in all the immunized animal groups in comparison control group. In case of IFN-γ (Figure 3B), a significant difference (*P<0.05; ***P<0.001) was noticed to all the immunized groups with respect to control except F1 group. No significant difference was noticed in the expression levels of IL-4 and IL-10 (Figure S2). Splenocytes from all groups responded to ConA non-specifically. The significant difference was observed in the expression level of IFN-γ (^#^P<0.001) in F1+LcrV+HSP70(II); LcrV+HSP70(II) and F1+HSP70(II) groups in comparison to F1+LcrV; LcrV and F1 groups respectively. The significant difference was observed in the expression level of IL-2 (^#^P<0.001) in F1+LcrV+HSP70(II) and LcrV+HSP70(II) groups in comparison to F1+LcrV; LcrV groups respectively. In the case of TNF-α, a significant difference (^#^P<0.001) was observed in F1+LcrV+HSP70(II) group in comparison to F1+LcrV group. The expression level of cytokines (IL-2, IL-4, IL-10, IFN-γ and TNF-α) in animal groups have been shown in Table 2.

**Figure 3:** Measurement of cytokines expressed by splenocytes of immunized mice groups. Cytokines expressed by splenocytes collected from mice immunized with F1, F1+HSP70(II), LcrV, LcrV+HSP70(II), F1+LcrV+HSP70(II) and HSP70(II) including control group were measured. Concentrations of cytokines detected in splenocytes supernatant after 48 h of stimulation with specific antigens (5 µg/ml) are shown. Graphs showed concentrations of (A) IL-2, (B) IFN-γ, (C) TNF-α in picograms per millilitre (pg/ml). Each bar represents the average of 8 mice/group ± S.D and is representative of three independent experiments. Analysis was done by one way ANOVA, All Pairwise Multiple Comparison Procedure (Fisher LSD Method). *P<0.05; **P<0.01; ***P<0.001; ^#^P<0.001.

**Table 2:** Expression level of cytokines in different animal groups.

S.N.	Groups	IL-2 (pg/ml)	IFN-γ (pg/ml)	TNF-α (pg/ml)	IL-4 (pg/ml)	IL-10 (pg/ml)
1.	Control	6.66±0.40	445.22±68.64	53±2.61	52.5±4.56	132.47±22.5
2.	F1	24.11±0.47	621.07±107.1	201.66±13.03	34.79±0.58	130.89±4.93
3.	F1+HSP70(II)	33.62±2.21	1344.82±127.67	267.06±12	30.15±1.05	144.58±4.93
4.	LcrV	52.5±2.46	761.86±82.5	553.77±42.92	32.16±1.69	203.78±20.51
5.	LcrV+HSP70(II)	96.61±1.69	1533.29±151.41	596.86±50	50.27±1.49	238.74±16.57
6.	F1+LcrV	70.68±0.85	965.85±110.76	620.12±15.98	54.75±3.07	255.77±23.14
7.	F1+LcrV+HSP70(II)	131.9±4.9	1761.63±122.34	794.27±90.79	55.25±1.09	250.38±12.18
8.	HSP70(II)	77.89±2.9	1165.72±310.45	710.93±105.83	54.41±2.73	239.71±6.54

RETRACTED

#### Enumeration of IFN-γ secreting CD4^+^ and CD8^+^ T cells by FACS

FACS analysis was performed for CD4+ and CD8+ T cell population producing IFN-γ in the splenocytes of all the immunized animal groups including control group. After stimulating splenocytes with specific antigen/s, an increased percentage of CD4^+^ T (Figure 4A) and CD8^+^ T cells expressing IFN-γ (Figure 5A) was observed in all vaccinated groups in comparison to control group. The population count (%) of IFN-γ secreting CD4+ T cells for Control, F1, F1+HSP70(II), LcrV, LcrV+HSP70(II), F1+LcrV, F1+LcrV+HSP70(II) and HSP70(II) groups was 0.46±0.12, 1.75±0.23, 1.16±0.12, 0.925±0.1, 0.98±0.12, 2.48±0.02, 4.43±0.52 and 4.985±0.04 respectively. The population count (%) of IFN-γ secreting CD4+ T cells for Control, F1, F1+HSP70(II), LcrV, LcrV+HSP70(II), F1+LcrV, F1+LcrV+HSP70(II) and HSP70(II) groups was 0.535±0.06, 1.17±0.04, 1.125±0.16, 0.91±0.43, 1.38±0.19, 2.725±0.99, 4.42±0.11 and 1.84±0.14 respectively. As shown by graphical representations, a significant difference (*P<0.05; **P<0.01; ***P<0.001) was noticed in the IFN-γ secreting CD4^+^ T cells (Figure 4B) and CD8^+^ T cells (Figure 5B) to all the immunized groups in comparison to control group. We also noticed a remarkable significant difference (^#^P<0.001) for both CD4+ and CD8+ T cells in F1+LcrV+HSP70(II) group in comparison to F1+LcrV group.

**Figure 4:** Flow cytometric analysis showing the percentage of IFN-γ producing CD4+ T cells in the spleens of immunized Balb/C mice following *in vitro* stimulation with specific antigens as indicated and anti-CD28 [A]. Graphical representation showing the significant difference in the percentage of IFN-γ producing CD4+ T cells in the spleen of different immunized animal groups after stimulation with specific antigens in comparison to the PBS control group. Each bar represents the average of 3 mice/group ± S.D [B]. Analysis was done by one way ANOVA, All Pairwise Multiple Comparison Procedure (Fisher LSD Method). **P<0.01; ***P<0.001; ^#^P<0.001.

**Figure 5:** Flow cytometric analysis showing the percentage of IFN-γ producing CD8+ T cells in the spleens of immunized Balb/C mice following *in vitro* stimulation with specific antigens as indicated and anti-CD28 [A]. Graphical representation showing the significant difference in the percentage of IFN-γ producing CD8+ T cells in the spleen of different immunized animal groups after stimulation with specific antigens in comparison to the PBS control group. Each bar represents the average of 3 mice/group ± S.D [B]. Analysis was done by one way ANOVA, All Pairwise Multiple Comparison Procedure (Fisher LSD Method). *P<0.05; **P<0.01; ***P<0.001; ^#^P<0.001.

RETRACTED

### Protection of immunized mice against intraperitoneal challenge with virulent *Y. pestis*

In order to compare the protective efficacy, the immunized animals were challenged with 100 LD_50_ of virulent *Y. pestis* including control group. Survivals of the animals were monitored for 30 days post challenge (Figure 6). Three vaccine combinations [LcrV+HSP70(II), F1+HSP70(II), F1+LcrV+HSP70(II)] resulted in 100% protection from the *Y. pestis* challenged mice (P<0.0001), whereas the LcrV and F1+HSP70(II) vaccinated mice were only 75% (P<0.001) and 12.5% protected, respectively. There was no protection observed in control, HSP70(II) and F1 groups. *Y. pestis* was recovered from the spleen, lung, liver and kidney of dead animals which succumbed to the challenge and identified by the growth on blood agar. Survived animals were sacrificed 30 days post-challenge, and autopsied for any bacterial presence in their organs like spleen, lung, liver and kidney. Vaccinated animals that survived the challenge appeared to clear *Y. pestis* from the mice since no growth was observed on blood agar plates from spleens, lungs, livers, and kidneys.

**Figure 6:** Determination of survival of Balb/C mice infected with *Y. pestis*. The immunized and PBS control groups (8 mice/group) were challenged with 100 LD_50_ of *Y. pestis* (S1 strain). The protective efficacy of vaccine candidate alone or in mixture of antigens was determined by Kaplan Meier's method to compare percentage survivals (****P<0.0001, ***P<0.001).

### Histopathological observations following *Y. pestis* infection

On day 3 and 20 after challenge with virulent *Y. pestis* (S1 strain), the lung, liver, kidney and spleen of the immunized groups including control group were isolated, fixed and prepared for HE staining. Normal mice that were neither immunized with plague vaccines or PBS nor infected with *Y. pestis* were used as naive controls.

The animals sacrificed on day 3 after infection, histopathological lesions were observed in the lung tissues (Figure 7a). Normal alveolar pattern with normal alveolar septa, air duct, alveoli and bronchioles with intact epithelium were observed from naive control group (Figure 7a [A]) whereas all the vaccinated including control group, lung parenchyma showed inflammation including neutrophil infiltration into the airways and alveoli as shown by arrow (Figure 7a [B]). The significant lung lesions were congestion, hemorrhage, granulovacuolar degeneration of bronchiole associated lymphoid tissue, bronchial lumen occlusion and psuedomembrane formation (Figure 7a [B-I]). Survived animals from LcrV; LcrV+HSP70(II); F1+LcrV and F1+LcrV+HSP70(II) vaccinated groups effectively recovered as no histopathological lesions were observed (Figure 7a [J-M]).

RETRACTED

**Figure 7:** Histopathology of the organs collected from the immunized group animals on 3^rd^ and 20^th^ day post infection with *Y. pestis* and the naive control animals that were neither immunized nor challenged with *Y. pestis*. Tissue sections were stained with hematoxylin and eosin for pathological examination. Tissue section collected from naive control and immunized animals on 3^rd^ day post infection *i.e.*, Naive control (A); PBS control (B); HSP70(II) (C); F1 (D); F1+HSP70(II) (E); LcrV (F); LcrV+HSP70(II) (G); F1+LcrV (H); F1+LcrV+HSP70(II) (I). Tissue sections were collected from the survived animal groups on 20^th^ day post infection *i.e.*, LcrV (J); LcrV+HSP70(II) (K); F1+LcrV (L); F1+LcrV+HSP70(II) (M). Photomicrograph represents the histopathology of Lung[**a**]: the arrows in the panel B indicate the infiltration of neutrophils. Photomicrograph of spleen [**b**]: in the panel B, reduced density of white pulp follicle and congestion in the red pulp, lymphoid follicle depletion shown by arrow and the presence of megakaryocytes shown by bold arrow. Photomicrograph of kidney [**c**]: the granular degeneration of parenchyma was observed in the panel B (bold arrows) and swelling in renal tubules (arrows). Photomicrograph of liver [**d**]: in the panel B, the hepatocytes degeneration was observed as indicated by arrow.

In spleen (Figure 7b), normal architecture with white pulp consisting of lymphatic follicles and red pulp consisting of sinusoidal and other element of blood were observed from naive control mice (Figure 7b [A]) whereas all the vaccinated animals including control group showed reduced density of white pulp follicles and congestion in the red pulp, lymphoid follicle depletion (arrow), lacking of lymphocytes, exhibiting higher number of myeloid and erythroid lineage cells and also presence of megakaryocytes as shown by bold arrow (Figure 7b [B-I]). Survived animals from LcrV; LcrV+HSP70(II); F1+LcrV and F1+LcrV+HSP70(II) vaccinated groups showed regression of splenic lesions except LcrV group that offered less protection and few megakaryocytes were seen (Figure 7b [J-M]).

RETRACTED

In kidney (Figure 7c), normal glomerulus, Bowman's space and renal parenchyma were observed from naive control mice (Figure 7c [A]) whereas the vaccinated and control group showed parenchymal granular degeneration (bold arrow), fragmentation of the chromatin material and renal tubule showing cloudy swelling with hydropic degeneration shown by arrow (Figure 7c [B-I]). Survived animals from LcrV; LcrV+HSP70(II); F1+LcrV and F1+LcrV+HSP70(II) vaccinated groups restored the normal appearance of renal capsule, glomeruli and renal tubules (Figure 7c [J-M]).

In liver (Figure 7d), normal hepatic cord arrangement, hepatic lobes and hepatocytes with normal hepatic parenchyma were observed in naive control mice (Figure 7d [A]) whereas vaccinated and control groups, liver histology exhibited granulovacuolar degeneration of hepatocytes (arrow), perinuclear clumping of the cytoplasm and obliteration of the chromatin material, few periportal and intraparenchymal small aggregates of macrophages and neutophils were seen (Figure 7d [B-I]). Survived animals from LcrV; LcrV+HSP70(II); F1+LcrV and F1+LcrV+HSP70(II) vaccinated groups recovered hepatic lesions, less infiltration of mononuclear cells and vacuolar degeneration (Figure 7d [J-M]).

### Localization of *Y. pestis* within infected animal tissues

To study the dissemination of *Y. pestis* from peritoneal cavity to various vital organs *i.e.*, lung, spleen, liver and kidney by immunohistochemistry were performed. The immunized animals including PBS control were sacrificed on day 3 after infection to localize *Y. pestis* by immunohistochemistry in lung, spleen, liver and kidney (Figure 8). No bacterium was observed in lung, liver, spleen and kidney isolated from the naive control group where as the clumping of *Y. pestis* was observed from all the vaccinated animals including control group by immunohistochemistry (Figure 8). On day 20 after infection, survived animals from LcrV; LcrV+HSP70(II); F1+LcrV and F1+LcrV+HSP70(II) groups were sacrificed for bacterial localization. No bacterial presence was observed in any of the survivors by immunohistochemistry (Fig. 8).

**Figure 8:** Immunohistochemistry (IHC) staining for localization of *Y. pestis* in the organs collected from immunized group animals on 3^rd^ and 20^th^ day post infection with *Y. pestis* and the naive control animals that were neither immunized nor challenged. The F1 antigen of *Y. pestis* was identified with anti-mouse FITC conjugated secondary antibody in the tissue sections collected from immunized animal groups on 3^rd^ day post infection including naive control *i.e.*, Naive control (A); PBS control (B); HSP70(II) (C); F1 (D); F1+HSP70(II) (E); LcrV (F); LcrV+HSP70(II) (G); F1+LcrV (H); F1+LcrV+HSP70(II) (I). Tissue sections were collected from the survived animal groups on 20^th^ day post infection *i.e.*, LcrV (J); LcrV+HSP70(II) (K); F1+LcrV (L); F1+LcrV+HSP70(II) (M). Fluorescent images representing the localization of *Y. pestis* in tissue sections of Lung [**a**]; Spleen [**b**]; Kidney [**c**]; and Liver [**d**].

RETRACTED

## Discussion

*Y. pestis* suppresses the host immune system in susceptible animal species, but the infection survived animals can effectively overcome the re-infection. This hints the possibility of developing effective vaccine that can boost the immune defense mechanisms against plague. Although intensive studies are in progress for several decades on plague [46] there is no safe and efficient vaccine till date. The F1/V based subunit vaccine candidate that evokes mainly humoral immune response, although has shown promising results in animal models, its efficacy in humans is not yet evaluated [47]. Further, the next-generation plague vaccines that are yet to be developed should also evoke cell-mediated immune response [28]. Humoral and cellular immunity potentially contribute to vaccine efficacy [48]. Humoral immunity relies upon production of antibodies by plasma B cells which effectively neutralizes extracellular pathogens while cellular immunity relies upon cytokine-producing capacities of T cells and is particularly effective in eradicating intracellular pathogens [49].

The protection evoked by cell-mediated immune response against intracellular pathogens mainly relies on Th1 type of immune response, considered by the development of pathogen-derived antigen specific IFN-γ and TNF-α secreting T cells [50], [51]. The *Y. pestis* replicates in macrophages of host and has developed a competent mechanism for the depletion of the NK cells that finally decreasing IFN-γ expression. The IFN-γ suppression obliterates the inflammatory response that is responsible for development of adaptive immunity [52]. It has been proved that STAT4-deficient mice with low level of IFN-γ were showing inadequate protection against *Y. pestis* infection despite producing high IgG antibody titers [53]. These findings indicate that high IgG titers may not be sufficient for vaccine efficacy. In case of plague, to develop an effective vaccine should evoke both humoral as well as strong Th1 type of cellular immune responses. Th1 type of immunity can assist to evoke the humoral immune response and to produce the long term memory cells. *In vivo* experiments proved that the administration of IFN-γ and TNF-α provide protection to mice against virulent *Y. pestis* challenge [54]. These evidences suggest that cellular immunity priming *Y. pestis* antigen specific Th1 CD4^+^ T cell is important for protection against plague.

RETRACTED

It is quite evident from the earlier studies that heat shock proteins (HSPs) are known to elicit potent T-cell responses not only to model antigens [31], [55] but also to the pathogen-derived antigens [35], [56]. HSP70(II) of *M. tuberculosis* is one of the examples to these various antigens, has been proven to evoke the T-cell response by several groups [31], [35], [55]. Ovalbumin-HSP70(II) (domain II) fusion constructs elicit ovalbumin-specific CD8+ cytotoxic T lymphocytes [36]. It has been demonstrated by Suzue and Young in 1996 that HSP70(II) of *M. tuberculosis* enhance the humoral and cellular immune response to the p24 protein of HIV1 [30].

In the present study, we evaluated three recombinant proteins F1, LcrV from *Y. pestis* and HSP70(II) (domain II) from *M. tuberculosis*. In order to augment the immune responses, HSP70(II) was formulated with F1 and LcrV and the animals were immunized with different combinations of antigen/s in formulation with aluminium hydroxide gel, a human compatible adjuvant. Sera from mice immunized with LcrV; LcrV+HSP70(II); F1+LcrV; F1+LcrV+HSP70(II) group had higher LcrV-specific IgG titers in comparison to F1-specific IgG titers in F1; F1+HSP70(II); F1+LcrV and F1+LcrV+HSP70(II) groups. HSP70(II) significantly induced high F1 and LcrV-specific serum IgG titers in F1+HSP70(II); LcrV+HSP70(II) and F1+LcrV+HSP70(II) immunized groups in comparison to F1, LcrV and F1+LcrV groups respectively. There are four IgG subclasses *viz*; IgG1, IgG2a, IgG2b, and IgG3 to provide the immunity against most of the infectious agents. In cell-mediated immune response, there is a change in the predominant immunoglobulin class or classes of the specific antibody produced. T-cells and their cytokines are mainly responsible to control the switch of these isotypes.

Th1 type of immune response signals via STAT4 to produce cytokines such as IFN-γ and IL-2 to favour a strong cellular immunity, whereas IL-4 signals via STAT-6 to favour a humoral immune response and thus biased towards Th2 type of immune response [53]. In this study, we observed significantly high level of Th1 type of cytokines *i.e.*, IL-2, IFN-γ and TNF-α in the splenocytes from all the vaccinated groups upon *in vitro* stimulation with group specific antigen/s in comparison to control group. HSP70(II) significantly modulated the expression level of IFN-γ in F1+HSP70(II); LcrV+HSP70(II) and F1+LcrV+HSP70(II) immunized groups in comparison to F1, LcrV and F1+LcrV groups respectively. In case of IL-2, a significant difference was observed in LcrV+HSP70(II) and F1+LcrV+HSP70(II) in comparison to LcrV and F1+LcrV groups respectively whereas TNF-α was observed in F1+LcrV+HSP70(II) group in comparison to F1+LcrV group. No significant difference in the expression level of Th2 type of cytokines (IL-4 and IL-10) was noticed. CD4^+^ T cells play an important role in the development of cellular immune responses and maintenance of memory CD8^+^ T cell responses [57]. The roles for CD8^+^ T cells during *Y. pestis* infection is not yet clear, but *Y. pestis* maintains virulence in the host by suppressing the production of Th1 type of cytokines [58]. Here, IFN-γ secreting CD4^+^ and CD8^+^ T cells were enumerated by flow cytometric analysis. A significant difference was observed in IFN-γ secreting CD4^+^ and CD8^+^ T cells in all vaccinated groups in comparison to control group. HSP70(II) significantly increased the IFN-γ secreting CD4^+^ and CD8^+^ T cells in F1+LcrV+HSP70(II) immunized group in comparison to F1+LcrV group.

RETRACTED

Histopathological assessment is valuable for evaluating the efficacy of new plague vaccines and for better understanding of the pathogenesis of the disease progression. To investigate whether the F1, LcrV and HSP70(II) antigens alone or in combination can effectively protect immunized animals from any histopathological alterations. Signs of histopathological lesions were noticed in lung, liver, kidney and spleen of immunized animals on 3^rd^ day post challenge. To examine the histopathological changes in survived animals of LcrV; LcrV+HSP70(II); F1+LcrV and F1+LcrV+HSP70(II) groups, three animals from each group were sacrificed on 20^th^ day post infection. The survived animals did not display any histopathological lesions in all the examined tissues. Immunohistochemistry showed bacteria in lung, liver, spleen and kidney on 3^rd^ day post infection whereas no bacterium was observed on 20^th^ day post infection in survived animals of LcrV, LcrV+HSP70(II), F1+LcrV and F1+LcrV+HSP70(II) vaccinated groups.

Several lines of evidence suggest that the outer surface proteins F1 and LcrV of *Y. pestis* are considered as the leading vaccine candidates and have been formulated to develop a subunit plague vaccine in the recent past [59]–[61],[48]. F1+LcrV combination can fully protect rodent models against lethal *Y. pestis* challenge [47], [62] however these vaccines provide poor and inconsistent protection (between 0 and 75%) in African Green monkeys [16]. Although these antigens are poorly immunogenic however their immunogenicity could be enhanced in formulation with Alum adjuvant [58] or by making a fusion protein with a molecular adjuvant like flagellin [63]. In this study, F1 and LcrV antigens have been formulated with HSP70(II) as an immunomodulator to augment the immune response of these two vaccine candidates. In mouse model, LcrV alone provided 75% protection whereas LcrV+HSP70(II) formulation provided 100% protection. F1 alone completely failed to protect whereas F1+HSP70(II) provided 12.5% protection. F1+LcrV and F1+LcrV+HSP70(II) provided 100% protection. Our finding proved that HSP70(II) enhanced the protective potential of F1 and LcrV vaccine candidates in mouse model however these formulations need to be tested in non human primates.

RETRACTED

## Supporting Information

Figure S1 Western blot analysis showing the reactivity of F1, LcrV and HSP70(II) with anti-F1[**A**], anti-LcrV[**B**] and anti-HSP70(II)[**C**] antibody respectively. The purified antigens F1, LcrV and HSP70(II) were run on SDS-PAGE and transferred to nitrocellulose membrane. F1, LcrV and HSP70(II) were recognized with their corresponding IgG antibody. The arrows on the right of the panels indicate the position of F1, LcrV and HSP70(II) protein bands.
(TIF)

Figure S2 Measurement of cytokines expressed by splenocytes of immunized mice groups. Cytokines expressed by splenocytes collected from mice immunized with F1, F1+HSP70, LcrV, LcrV+HSP70, F1+LcrV+HSP70 and HSP70 including control group were measured. Concentrations of cytokines detected in splenocytes supernatant after 48 h of stimulation with specific antigens (5 µg/ml) are shown. Graphs showed concentrations of IL-4 [A] and IL-10 [B] in pg/ml. Each bar represents the average of 8 mice/group ± S.D and is representative of three independent experiments. Analysis was done by one way ANOVA, All Pairwise Multiple Comparison Procedure (Fisher LSD Method). No significant difference was observed.
(TIF)
